# Clinical Application of a Modified Double Purse-String Continuous Suture Technique for Pancreaticojejunostomy: Reliable for Laparoscopic Surgery and Small Size Main Pancreatic Duct

**DOI:** 10.1155/2021/6676999

**Published:** 2021-03-13

**Authors:** Delin Ma, Gang Du, Jinhuan Yang, Jianping Song, Huan Ma, Jianlei Wang, Tingxiao Zhang, Bin Jin

**Affiliations:** Department of General Surgery, Qilu Hospital, Shandong University, No. 107, Wenhua Xi Road, Jinan 250012, China

## Abstract

**Background:**

The technical challenge of pancreatojejunostomy (PJ) is the greatest barrier for surgeons to complete pancreatoduodenectomy (PD). The authors present an easy-to-master PJ anastomosis technique with limited technical requirements. This technique uses two layers of sutures and double purse-string sutures to complete the entire anastomosis. This anastomosis technique has achieved good results in laparoscopic surgery (LS) and small size main pancreatic duct (MPD).

**Methods:**

From February 2015 to August 2020, 63 patients who met the surgical indications underwent a modified double purse-string continuous suture pancreaticojejunostomy technique in our center. We collected patient demographic characteristics and perioperative outcomes and analyzed these data.

**Results:**

A total of 63 patients underwent PD using our new anastomosis technique. Thirty-eight patients underwent LS, and 26 patients had a small MPD (<3 mm). The median operative time (OT) was 270 min, and the median estimated blood loss (EBL) was 200 ml. Ten patients had grade B postoperative pancreatic fistula (POPF), while no patients had grade C POPF. No 90-day mortality was observed. There were significant differences in the OT and postoperative hospital stay (PHS) among groups with different surgical procedures, while there were no significant differences among groups with different MPD sizes. Neither the surgical procedure nor the MPD size affected early postoperative complications.

**Conclusion:**

This new technique can not only reduce the incidence of POPF but also is reliable for LS and surgeries with small size MPD. Therefore, this technique is worthy of clinical promotion and application in the future.

## 1. Introduction

Pancreaticoduodenectomy (PD), first reported by Walther Kausch in 1909 [1], has been universally recognized as the only radical treatment for patients with cancer of the lower bile duct, papillary duodenum, periampullary ampulla, and head of the pancreas since its emergence. However, due to the challenges of extensive visceral organ dissection and complicated digestive tract reconstruction, PD is considered one of the most complex gastrointestinal surgical operations. Especially in LS, restricted by the operation angle and the length of the instrument, the difficulty of laparoscopic suturing and knotting is significantly increased, which makes PD further complicated. Furthermore, as the most critical step of PD, the quality of pancreaticojejunostomy (PJ) is of great significance as that determines the incidence of anastomotic complications, especially postoperative pancreatic fistula (POPF) [2, 3]. To reduce the incidence of POPF, various reconstruction methods have also been developed to diminish pancreatic leakage, such as the duct-to-mucosa technique, the invagination technique, and their modifications [4, 5]. However, there is still no ideal way to significantly reduce the risk of POPF. After a long period of exploration, we put forward a modified double purse-string continuous suture pancreaticojejunostomy technique, which is characterized by its simple operation and reasonable procedure. After clinical applications in recent years, its effect has proven to be reliable.

## 2. Materials and Methods

### 2.1. Inclusion Criteria of Patients

Between February 2015 and August 2020, 63 patients who underwent PD with this modified double purse-string continuous suture pancreaticojejunostomy technique at Qilu Hospital of Shandong University in Jinan (China) were enrolled in this study. The inclusion criteria for the patients are as follows: (1) older than 20 years and younger than 85 years of age, (2) generally in good condition, without contraindications for general anesthesia or surgery, and (3) with a resectable tumor (without macrovascular invasion or vital organ invasion or any evidence of metastasis in any other site).

### 2.2. Preoperative Preparation

All patients met the surgical requirements. They received adequate preoperative preparation, including respiratory exercises, correction of water electrolyte and acid-based imbalance, and control of blood sugar and blood pressure. In addition, for patients who had apparent obstructive jaundice (total serum bilirubin level > 200 *μ*mol/l), our center preferentially used percutaneous transhepaticcholangial drainage (PTCD) to reduce the jaundice. On the day before the operation, all patients and their families were informed in advance of the operation details and risks, and the informed consent forms were signed. This study received ethical approval from the Ethics Committee of Qilu Hospital at Shandong University (approval number: KYLL-202011-180).

### 2.3. Data Collection

The demographic characteristics and perioperative outcomes of all patients were collected from the electronic clinical data system in our hospital. The data included age, sex, body mass index (BMI), preoperative comorbidities, history of smoking, history of alcohol consumption, history of abdominal surgery, pathology data, tumor size, main pancreatic duct (MPD) size, surgical procedure, operative time (OT), estimated blood loss (EBL), intraoperative transfusion, postoperative transfusion, days of postoperative transfusion, days of indwelling gastric tube use, blood transfusion, postoperative complications, days of postoperative hospital stay (PHS), and 90-day mortality. We then further divided patients into subgroups according to their surgical type and the MPD size. The demographic characteristics and perioperative outcomes were analyzed for each subgroup.

### 2.4. Definition of Postoperative Complications

Postoperative complications were graded according to the Clavien-Dindo ranking system [6]. The diagnosis and grade of POPF were determined according to the criteria of the International Study Group on Pancreatic Fistula (ISGPF) [7]. Original grade A POPF was no longer considered as a true pancreatic fistula, and it was renamed as a biochemical fistula. When a change was needed in the management of the expected postoperative pathway, grade B could be diagnosed. Whenever a grade B POPF led to organ failure or to clinical instability such that reoperation was needed, POPF became grade C. Delayed gastric emptying was diagnosed according to a suggested definition by the International Study Group of Pancreatic Surgery (ISGPS) [8], and patients who reached grade B or higher of this criteria were defined as having delayed gastric emptying. Bile leakage was defined as the abdominal drainage fluid having any amount of bile and/or the presence of bilirubin levels >3 times the serum bilirubin levels [9]. Cardiac events included acute coronary syndromes and cardiac failure, while respiratory events included respiratory insufficiencies requiring invasive organ support and pneumonia.

### 2.5. Surgical Technique

PD was performed using the standard procedure, and sites of visceral resection included the pancreatic head, pancreatic neck, distal stomach, duodenum, proximal jejunum, gallbladder, and common biliary duct. The Standard-Child reconstruction, i.e., using one single jejunal loop to connect the pancreas and biliary anastomosis with the gastrojejunostomy, was subsequently performed for digestive tract reconstruction [10].

#### 2.5.1. PJ Surgical Technique

*(1) Management of the Pancreatic Stump*. The pancreatic parenchyma containing the tumor was carefully excised with an ultrasonic scalpel. During this procedure, care was taken to avoid injuring the MPD. Then, full hemostasis of the pancreatic cut surface was achieved using electrocoagulation or an ultrasonic scalpel. Next, the pancreatic stump was freely dissected by approximately 1-2 cm in length from the splenic artery and vein to facilitate anastomosis. According to the diameter of the MPD, a support tube with a diameter corresponding to the MPD was selected and inserted as the internal stent (Figures 1(a) and 2(a)). We made several holes in the support tube at different positions. The purpose of this step was to ensure uninhibited outflow of pancreatic fluid. The length of the support tube outside the pancreas was maintained at 5-6 cm. The proximal segment of the jejunum was moved to the bed of the resected duodenum to facilitate subsequent surgical procedures.

*(2) Purse-String Suturing at the Pancreatic Stump*. Purse-string suturing at the pancreatic stump was executed by using 4-0 nonabsorbable sutures (Prolene; Ethicon, Inc., NJ). The detailed steps are as follows. The suture was placed starting from the pancreatic parenchyma, after which the needle was passed transversally through the support tube and was finally passed again through the pancreatic parenchyma. The entry and exit points of the needle should stay at least 3 mm away from the MPD to prevent tearing of the tissue (Figures 1(b) and 2(b)). Next, we employed the purse-string suturing technique around the MPD in a clockwise or counterclockwise direction, and the suture was tied after the procedure was completed (Figures 1(c) and 2(c)).

*(3) Suturing the Posterior Layer of the Anastomosis*. The posterior layer of the anastomosis was initiated from the posterosuperior side of the pancreatic cut surface. The first stitch should traverse the pancreas in full thickness from anterior to posterior. The entry and exit points of this stitch should had a distance of 0.5-1 cm from the cut surface of the pancreas. Subsequently, from superior to inferior, we used 4–0 nonabsorbable sutures (Prolene; Ethicon, Inc., NJ) to perform continuous suturing between the pancreatic parenchyma and the seromuscular layer of the jejunum. The sutures were not immediately tightened; rather, they were allowed to remain a few centimeters apart to facilitate exposure for the next several stitches (Figures 1(d) and 2(d)). In addition, the distance between the entry and exit points on the jejunal wall was wide enough to allow the jejunal wall to wrap the pancreatic stump after the sutures were tightened. The requirements of the last stitch were identical to those of the first stitch, which needed to traverse the pancreas in full thickness from anterior to posterior. Finally, the sutures were tightened and tied gently to approximate the pancreatic stump and the jejunum limb via parachuting without laceration or ischemia of the pancreatic parenchyma.

*(4) Purse-String Suturing at the Jejunal Wall*. We made a small hole on the jejunal wall opposite the MPD with an ultrasonic scalpel. The free end of the MPD stent was passed through this hole into the enteric cavity. Next, a 4-0 nonabsorbable suture (Prolene; Ethicon, Inc., NJ) was inserted from the anterior pancreatic stump and pierced out from the back of the support tube. Subsequently, we executed purse-string suturing around the small hole on the jejunal wall. The suture was again passed through from the back of the support tube, penetrated the pancreatic parenchyma, and finally pierced out from the anterior pancreatic stump. After the above steps, two sutures crossed each other behind the stent, thereby forming a shape similar to a figure eight (Figures 3(a) and 2(e) and (f)). Finally, it was tightened and tied.

*(5) Suturing the Anterior Layer of the Anastomosis*. We performed continuous suturing between the anterior transected surface of the pancreas and the seromuscular layer of the jejunum. The technical details were similar to those described in the posterior layer (Figures 3(b) and 2(g)). Immediately after, the gap between the pancreatic stump and the jejunum limb was closed by tightening the suture (Figures 3(c) and 2(h)). Depending on the situation, the superior and inferior edges of the pancreatic stump could be sutured individually, with the aim of wrapping the jejunum around the superior and inferior edges of the pancreatic stump.

#### 2.5.2. The Remaining Digestive Tract Reconstruction

Choledochojejunostomy was performed at a distance of 10 cm downstream of the PJ. Next, gastroenterostomy was finished at a distance of approximately 50 cm from the choledochojejunostomy. Finally, the operating fields were inspected carefully for active bleeding. After no bleeding was confirmed, we placed drainage tubes, sutured the incision, and finished the operation.

### 2.6. Statistical Analysis

Data processing was conducted using SPSS version 25.0 software (SPSS Inc., Chicago, Illinois, USA). Normally, distributed continuous data are expressed as the mean ± standard deviation (SD), while non-normally distributed continuous data are expressed as the median and interquartile range (IQR). Student's *t*-tests or Mann–Whitney *U*-tests were used to compare the variables according to their distributions. Categorical data are expressed as numbers and percentages, and chi-square tests or Fisher's exact tests were used for these data. A *P* value less than 0.05 was considered statistically significant.

## 3. Results

### 3.1. Patient Characteristics

The demographic and pathological characteristics of the patients are summarized in Table 1. In this study, 44 men and 19 women were recruited with a mean age of 60.4 years. The average BMI was 23.1 kg/m^2^. In terms of comorbidities, 10 patients (15.9%) had diabetes, 16 (25.4%) patients had hypertension, and 3 patients (4.8%) had coronary heart disease. In addition, twenty-nine (46.0%) out of the 63 patients had a history of smoking, and 32 (50.8%) had a history of alcohol consumption. Ten patients (15.9%) had a history of abdominal surgery. The most common histologic type was distal cholangiocarcinoma, followed by pancreatic ductal adenocarcinoma. The median tumor size was 2.5 cm. There were 26 patients (41.3%) that had a small MPD size with diameter < 3 mm. Thirty-eight (60.3%) patients underwent LS, while 25 patients (39.7%) underwent OS in our study.

### 3.2. Perioperative Outcomes

The perioperative outcomes are summarized in Table 2. The median OT was 270 min, and the median EBL was 200 min. Intraoperative transfusion occurred in 1 patient, and postoperative transfusion occurred in 16 patients (25.4%). The median postoperative defecation time was 2 days, and the median time of indwelling gastric tube use was 7 days. Forty-four patients (69.8%) suffered from early postoperative complications, while 9 of them (14.9%) were classified to Clavien-Dindo grade 3 and higher. According to the diagnostic criteria of ISGPF, 10 patients (15.9%) had grade B POPF, while no patients had grade C POPF. Twenty-six patients (41.3%) had delayed gastric emptying, and all of these patients recovered with conservative therapy. In addition, 7 patients (11.1%) experienced postoperative hemorrhage. Among these, 2 accepted arterial embolization to achieve hemostasis, one was investigated by gastroscopy, and the rest were cured through conservative treatment. Other postoperative complications included respiratory events in 5 patients (7.9%), surgical wound infections in 3 patients (4.8%), bile leakage in 2 patients (3.2%), abdominal infections in 1 patient (1.6%), and cardiac events in 1 patient (1.6%) These complications were controlled using conservative treatment without surgical intervention. The median time of PHS was 18 days. There was no 90-day mortality after the operation.

### 3.3. Clinical Outcomes according to the Surgical Procedure

The comparison between the OS (*n* = 25) and LS (*n* = 38) groups is summarized in Table 3. There was no significant difference between the two groups in terms of demographics, tumor size, or main pancreatic duct size (Table 3, *P* > 0.05). Comparing the perioperative outcomes, the two groups had similar estimated blood loss, postoperative defecation, and indwelling gastric tube use (Table 3, *P* > 0.05). Although the rates of pancreatic fistula (Table 3, 24.0% vs. 10.5%, *P* > 0.05) and morbidity (Table 3, 76.0% vs. 65.8%, *P* > 0.05) were slightly higher in the OS group than in the LS group, this difference was not statistically significant. The LS group had a longer OT (Table 3, 305 vs. 220 min, *P* < 0.001) but shorter length of PHS (Table 3, 17.5 vs. 21 days, *P* = 0.012) than the OS group, and this difference was statistically significant.

### 3.4. Clinical Outcomes according to the MPD Size

The comparison between the two groups with different MPD sizes is summarized in Table 4. The demographics, tumor size, and MPD size were not significantly different (Table 4, *P* > 0.05), although the mean age in the LMPD group was slightly higher than that in the SMPD group (Table 4, 62.5 vs. 57.5 years, *P* = 0.044). At the same time, no statistically significant differences were found in the surgical procedures or conversion rates between the two groups (Table 4, *P* > 0.05). There were no significant differences between them with respect to the OT, EBL, postoperative transfusion rate, postoperative defecation, indwelling gastric tube use, morbidity rate, pancreatic fistula rate, or 90-day mortality rate (Table 4, *P* > 0.05).

## 4. Discussion

In recent years, with the deepened gradual understanding of pancreatic anatomy and the emergence of a series of new surgical instruments, LS has been greatly broadened. An increasing number of centers are now shifting towards LS. There are studies indicating that this approach also has significant advantages in terms of shortened hospital stay, fewer postoperative morbidities, and enhanced recovery [11–13]. However, LS is associated with several technical disadvantages, such as a lack of tactile sensation and a narrow visual field. This limitation is particularly evident in pancreatic surgery when performing PJ. If surgeons place excessive tension on sutures during tying, the pancreatic parenchyma may get torn. This could reduce the quality of PJ and increase the incidence of pancreatic fistula. In addition, the diameter of the MPD has strong association with the incidence of POPF [2, 3], because the MPD of most patients is not dilated and is too small to perform precise anastomosis. Here, we described an ideal anastomosis technique for PJ that is applicable and practical for both OS and LS regardless of the MPD size.

Toward this goal, we made several changes to improve our PJ. Considering the technical difficulty of laparoscopy, continuous sutures have more advantages in many aspects than interrupted sutures. First, running suturing between the pancreatic parenchyma and the jejunal wall is evenly distributed, which causes less damage to the pancreatic parenchyma. The gap between the pancreatic stump and the jejunal wall will be closed without leaving any dead space after the suture is tightened and ligated, which can prevent retention of pancreatic juice and effusion from the pancreatic stump. Furthermore, the suture was not tightened when suturing, and there was a certain distance between the pancreatic parenchyma and jejunum during the whole process. Therefore, the surgical field was clear, which facilitated the suture performance under laparoscopy and shortened the time needed for the anastomosis, thus shortening the whole operation time. In recent years, a number of studies have shown that continuous sutures have a lower risk of postoperative complications and POPF than interrupted sutures in both open and minimally invasive surgery [14–17]. Second, many surgeons tend to perform an inner layer of the anastomosis between the wall of the main pancreatic duct and the full layer of the jejunum [14, 18]. However, this procedure becomes very difficult and has a high risk of a full thickness tear of the MPD when performed laparoscopically or when the MPD is too small. Hence, we made a further modification by inserting a support tube sutured with double purse-string sutures to replace the inner layer of the anastomosis. The support tube can maintain alignment of the MPD with the small incision in the jejunal wall and prevent occlusion of the MPD during suturing. The double purse-string suture allows the wall of the MPD and the jejunal wall to be closer to the support tube, thus preventing pancreatic juice and intestinal contents from entering the anastomotic space. Furthermore, the second purse-string suture with a shape similar to a figure eight plays an important role in strengthening the inner layer of the anastomosis.

Once patients suffer from POPF, the worst complication after PD, especially grade B or C pancreatic fistula, a series of other severe morbidities or even mortality can develop. As this is closely related to the occurrence of pancreatic fistula, whether pancreatic anastomosis technology can reduce the incidence of pancreatic fistula is an important criterion to test its quality. In several large-volume studies using the updated POPF defined by the ISGPS in 2016 as the diagnostic criterion, the incidence of grade B/C pancreatic fistula was 18.5% to 33% [19–21]. In our study, this result was 15.9%, and no patients developed grade C pancreatic fistula. Another noteworthy feature of our study is that a large proportion of patients defined as having grade B pancreatic fistula were separated from the biochemical leakage group simply because the drainage tube had been placed for more than 21 days. In a previous study, researchers also found that the clinical impact in patients treated with persistent drain placement alone was similar to that in biochemical leakage patients [20]. These patients were often observed to have grade B POPF treated with conservative drainage; so, conservative drain management increased the incidence of grade B pancreatic fistula. Therefore, it is reasonable to believe that if we change our conservative drain management, we may have a lower incidence of grade B/C pancreatic fistula. Taken together, We believe that our modified double purse-string continuous suture pancreaticojejunostomy technique is safe and reliable.

Comparing the perioperative outcomes of the two different surgical groups, we found that the LS group was superior to the OS group in terms of PHS, while it was inferior to the OS group in terms of OT, which is similar to previous studies [21–24]. Several reasons may account for this marked difference. One possible reason for longer OT of LS is that LS lacks tactile feedback and makes the operation inconvenient. However, this can be improved by the accumulated surgical experience, and in our study, the last ten patients in the endoscopy group had shorter operative times than the first ten patients (305 vs. 358.5 min). The possible reason for better PHS of LS is that OS introduces bigger trauma and takes longer postoperative recovery. There was no significant difference in postoperative complications and the incidence of pancreatic fistula, which suggested that this anastomosis technique could achieve the same good results in both surgical procedures. In addition, our results were superior to those of a randomized controlled trial by Van Hilst et al. [21] in many aspects, such as shorter OT (305 vs 410 min in LS, 220 vs 274 min in OS), lower EBL (200 vs 300 ml in LS, 200 vs 450 ml in OS), lower morbidity rate with Clavien grade ≥ 3 (15.8% vs 50.0% in LS, 12.0% vs 39.0% in OS), and lower incidence of grade B/C pancreatic fistula (10.5% vs 28.0% in LS, 24.0% vs 24.0% in OS).

Surgeons are unable to design individualized plan tailored to the MPD size of these patients in practice. An ideal pancreatic anastomosis technique should be applicable regardless of the pancreatic duct size. To evaluate this effect, we further classified the patients according to MPD size and found that smaller MPD size did not affect the clinical outcomes, including OT, EBL, postoperative transfusion rate, postoperative defecation, indwelling gastric tube use, morbidity rate, pancreatic fistula rate, PHS, and 90-day mortality rate. These perioperative outcomes might suggest that the modified double purse-string continuous suture pancreaticojejunostomy technique is technically safe and reliable for patients even when the pancreatic duct is too small.

However, this study has some limitations. First, we did not do power calculation for this study and only analyzed the available patients in the database. We plan to update our results after accumulating more patients. Second, we did not obtain follow-up data of patients in our study that would provide more information of the surgery effects. Third, we did not have a control group that received other treatment modalities. The main purpose of this study was to describe our surgical technique, and the next step is to conduct a comparative study between different surgical techniques after accumulating enough cases, preferably in a high-quality prospective randomized environment, to conduct a multicenter experiment. In addition, similar to other retrospective study, there is a possibility of selection bias, data collection is limited to only the data that are available, and data such as time of PJ and pancreatic texture were not well documented in our database. Finally, all the operations were performed by one team which has rich experience in the field of PD. Therefore, we could not exclude the possibility that this acceptable result in our study may be due to the exquisite technique of the doctor, and it is necessary to conduct further multicenter research.

## 5. Conclusions

In general, according to the current results, we have proved that this modified double purse-string continuous suture technique pancreaticojejunostomy is a safe and reliable surgical method. It is highly suitable in both open surgery (OS) and laparoscopic surgery (LS). Moreover, this technique shows that good results can be achieved even in small main pancreatic ducts. To further validate the results, further prospective multicenter studies are necessary.

## Figures and Tables

**Figure 1:** Schematic diagram of PJ. (a) A schematic diagram of the pancreatic stump and the jejunal limb. (b) The needle penetrated the support tube. **(c)** A purse-string suture was placed on the pancreatic stump. (d) Continuous suturing was used to complete the posterior layer anastomosis.

**Figure 2:** Video screenshots of PJ under the laparoscope. (a). Management of the pancreatic stump. (b) The needle penetrated the support tube. (c) A purse-string suturing around the MPD was completed on the pancreatic stump. (d) The posterior layer of the anastomosis was completed. (e, f) A small hole was made on the jejunal limb, and the free end of the support tube was inserted into it. The purse-string suturing on the jejunal limb combining with intersecting sutures behind the stent formed a shape similar to a figure eight. (g) The anterior layer of the anastomosis was completed. (h) The whole anastomosis was completed.

**Figure 3:** Schematic diagram of PJ. (a) The posterior layer of the sutures was tightened, and the free end of the support tube was inserted into the hole. Then, purse-string suturing was completed on the jejunal limb. (b) The anterior layer of the anastomosis was completed. (c). The anterior layer of the sutures was tightened, and the whole anastomosis was completed. (d) A schematic diagram of the suturing of the whole anastomosis.

**Table 1:** Summary of patient demographic and pathological characteristics.

Variables	
Age, years	60.4 ± 9.8
Male, *n* (%)	44(69.8)
BMI^#^, kg/m^2^	23.1 ± 3.3
Comorbidities, *n* (%)	
Diabetes	10 (15.9)
Hypertension	16 (25.4)
Coronary heart disease	3 (4.8)
History of smoking, *n* (%)	29 (46.0)
History of alcohol consumption, *n* (%)	32 (50.8)
History of abdominal surgery, *n* (%)	10 (15.9)
Pathology, *n* (%)	
Distal cholangiocarcinoma	16 (25.4)
Pancreatic ductal adenocarcinoma	15 (23.8)
Duodenal adenocarcinoma	14 (22.2)
Carcinoma of Vaters ampulla	8 (12.7)
Pancreatic neuroendocrine tumor	3 (4.8)
Chronic pancreatitis	2 (3.2)
Hamartoma	2 (3.2)
Other pathological types^∗^	3 (4.8)
Tumor size, cm	2.5 (2-3)
Main pancreatic duct size, *n* (%)	
<3 mm	26 (41.3)
≥3 mm	37 (58.7)
Surgical procedure, *n* (%)	
Laparoscopic surgery	38 (60.3)
Open surgery	25 (39.7)

Data are presented as the mean with standard deviation (x ± SD) or counts with percentages (*x*%). #BMI: body mass index. ^∗^Other pathological types included intraductal papillary mucinous neoplasm in one case (1.6%), pancreatic cystadenoma in one case (1.6%), and duodenal stromal tumor in one case (1.6%).

**Table 2:** Summary of patient perioperative outcomes.

Variables	
Operative time, min	270 (225-335)
Estimated blood loss, ml	200 (150-200)
Intraoperative transfusion, *n* (%)	1 (1.6)
Postoperative transfusion, *n* (%)	16 (25.4)
Postoperative defecation, days	2 (2-4)
Indwelling gastric tube use, days	7 (5-9)
Morbidity, *n* (%)	44 (69.8)
Clavien 1–2	35 (55.6)
Clavien ≥3	9 (14.3)
Pancreatic fistula, *n* (%)	
Normal or biochemical leak	53 (84.1)
Grade B	10 (15.9)
Grade C	0 (0)
Other complications, *n* (%)	
Delayed gastric emptying	26 (41.3)
Postoperative hemorrhage	7 (11.1)
Respiratory events	5 (7.9)
Surgical wound infection	3 (4.8)
Bile leakage	2 (3.2)
Abdominal infection	1 (1.6)
Cardiac events	1 (1.6)
Postoperative hospital stay, days	18 (15-22)
90-day mortality, *n* (%)	0 (0)

Data are presented as the median with interquartile range (median [25%, 75%]) or counts with percentages (*x*%).

**Table 3:** Comparison between patients with laparoscopic surgery (LS group) and open surgery (OS group).

Variables	LS group (*n* = 38)	OS group (*n* = 25)	*P* value
Age, years	60.5 ± 10.7	60.4 ± 8.4	0.973
Male, *n* (%)	25 (65.8)	19 (76.0)	0.388
BMI^#^, kg/m^2^	22.6 ± 2.7	23.7 ± 3.9	0.205
Tumor size, cm	2.5 (1.95-3.5)	2.5 (1.9-3)	0.854
Main pancreatic duct size, *n* (%)			
<3 mm	14 (36.8)	12 (48.0)	0.379
≥3 mm	24 (63.2)	13 (52.0)	
Operative time, min	305 (265-358.75)	220 (197.5-242.5)	**<0.001**
Conversion rate^∗^, *n* (%)	5 (13.2)		
Estimated blood loss, ml	200 (200-200)	200 (125-200)	0.868
Postoperative transfusion, *n* (%)	10 (26.3)	6 (24.0)	0.836
Postoperative defecation, days	2 (1.75-4)	3 (2-4)	0.234
Indwelling gastric tube use, days	7 (5-9.25)	7 (6-9.5)	0.193
Morbidity, *n* (%)	25 (65.8)	19 (76.0)	0.388
Clavien 1–2	19 (50.0)	16 (64.0)	0.547
Clavien ≥3	6 (15.8)	3 (12.0)	
Pancreatic fistula, *n* (%)			
Normal or biochemical leak	34 (89.5)	19 (76.0)	0.176
Grade B	4 (10.5)	6 (24.0)	
Grade C	0 (0)	0 (0)	
Postoperative hospital stay, days	17.5 (14-20.25)	21 (16-26.5)	**0.012**
90-day mortality, *n* (%)	0 (0)	0 (0)	N/A

#BMI: body mass index. ^∗^Patients converted to open surgery are still included in the LS group for analysis. Data are presented as the mean with standard deviation (*x* ± SD) or median with interquartile range (median [25%, 75%]), or counts with percentages *n* (*x*%). Bold text indicates a statistically significant value.

**Table 4:** Comparison between patients with small (<3 mm, SMPD group) and large (≥3 mm, LMPD group) MPD.

Variables	SMPD group (*n* = 26)	LMPD group (*n* = 37)	*P* value
Age, years	57.5 ± 11.0	62.5 ± 8.4	**0.044**
Male, *n* (%)	16 (61.5)	28 (75.7)	0.229
BMI^#^, kg/m^2^	23.6 ± 3.6	22.7 ± 2.9	0.305
Tumor size, cm	2.5 (2-3.5)	2.5 (1.8-3)	0.280
Surgical procedure, *n* (%)			
Laparoscopic surgery	14 (53.8)	24 (64.9)	0.379
Open surgery	12 (46.2)	13 (35.1)	
Conversion rate, *n* (%)	1 (7.1)	4 (16.7)	0.633
Operative time, min	277.5 (225-351.25)	265 (225-315)	0.472
Estimated blood loss, ml	200 (200-225)	200 (125-200)	0.152
Postoperative transfusion, *n* (%)	5 (19.2)	11 (29.7)	0.346
Postoperative defecation, days	2 (2-4)	3 (2-3.5)	0.636
Indwelling gastric tube use, days	7 (5-10)	7 (6-9)	0.578
Morbidity, n (%)	17 (65.4)	27 (73)	0.518
Clavien 1–2	15 (57.7)	20 (54.1)	0.433
Clavien≥3	2 (7.7)	7 (18.9)	
Pancreatic fistula, *n* (%)			
Normal or biochemical leak	21 (80.8)	32 (86.5)	0.728
Grade B	5 (19.2)	5 (13.5)	
Grade C	0 (0)	0 (0)	
Postoperative hospital, days	20 (15-27)	18 (14-21)	0.085
90-day mortality, *n* (%)	0 (0)	0 (0)	N/A

MPD: main pancreatic duct; ^#^BMI: body mass index. Data are presented as the mean with standard deviation (*x* ± SD), or median with interquartile range (median [25%, 75%]) or counts with percentages *n* (*x*%). Bold text indicates a statistically significant value.

## Data Availability

The datasets used and/or analyzed during the current study are available from the corresponding author on reasonable request.

## Abbreviations

LS: Laparoscopic surgery
OS: Open surgery
PD: Pancreaticoduodenectomy
PJ: Pancreaticojejunostomy
PTCD: Percutaneous transhepaticcholangial drainage
BMI: Body mass index
MPD: Main pancreatic duct
OT: Operative time
EBL: Estimated blood loss
PHS: Postoperative hospital stay
ISGPF: International Study Group on Pancreatic Fistala
ISGPS: International Study Group of Pancreatic Surgery
SD: Standard deviation
IQR: Interquartile range.
